The article "Multislice Spiral Computed Tomography Postprocessing Technology in the Imaging Diagnosis of Extremities and Joints" was published in 2021. Journal: Comput Math Methods Med.

# Multislice Spiral Computed Tomography Postprocessing Technology in the Imaging Diagnosis of Extremities and Joints

**DOI:** 10.1155/2021/9533573

**Published:** 2021-12-13

**Authors:** Weihua Yang, Fei Wang

**Affiliations:** ^1^Xinxiang University, Xinxiang, Henan 453003, China; ^2^Hainan General Hospital, Haikou, Hainan 570311, China

## Abstract

**Objective:**

To improve the clinical detection rate of bone and joint fractures of the extremities and to explore the value and significance of the application of multislice spiral computed tomography (MSCT) postprocessing technology in diagnosis.

**Methods:**

80 patients with bone and joint fractures of the extremities admitted to the hospital were selected as the research objects. The patients received X-ray digital radiography (DR) plain film examination and then MSCT examination. At the same time, multiplane reconstruction (MPR) and surface shadow display (SSD) and volume rendering three-dimensional imaging (VRT) technology and other postprocessing technologies compare the differences in the detection rate of limbs and joint fractures between the two inspection methods.

**Results:**

A total of 100 fractures were found in 80 patients. The detection rate of X-ray DR was 69%. After MSCT postprocessing technology, the detection rates of MPR, SSD, and VRT were 96%, 98%, and 99%, respectively. The accuracy of MSCT postprocessing technology in diagnosing extremity bone and joint fractures was significantly higher than that of DR, and the difference between groups was statistically significant.

**Conclusion:**

MSCT postprocessing technology for patients with extremity bone and joint fractures has a good effect. It is not only noninvasive but also has a high detection rate. It can significantly reduce the missed and misdiagnosed rate and provide detailed imaging data for the formulation of clinical treatment plans.

## 1. Introduction

Bone and joint fractures of extremities are a common type of fracture in clinical practice, which seriously endanger the health of patients [1–3]. At present, many patients with extremity bone and joint fractures are diagnosed by X-ray film [4, 5] to determine whether the patient has extremity bone and joint fractures. X-ray examination is the first choice in clinical imaging. However, X-ray plain film examination has certain limitations for occult fractures. Suspicious fractures are prone to missed and misdiagnosed situations, which delays the clinical treatment of patients with limb bone and joint fractures.

The implementation of multilayer spiral computed tomography (MSCT) scanning and three-dimensional reconstruction technology for patients with extremity bone and joint fractures can help to quickly and accurately diagnose the damage of extremities and joints [6–9] and provide more detailed imaging data for the clinical treatment of patients. The effective use of multislice spiral CT postprocessing technology can establish three-dimensional images and intuitively feedback the images of the patient's limbs and joint fractures.

Fractures of the limbs and joints can easily affect the life and work of patients [10]. In the past, digital radiographs were mostly used in clinical examinations, but due to the overlap of structures, they can only observe the lesions from a single angle, and often fail to clearly show the lesions, leading to missed and misdiagnosed small or hidden fractures, which is not conducive to clinical guidance follow-up treatment. In addition, patients with limb bone and joint fractures are affected by factors such as pain and dysfunction during the filming, and the position of the film is not accurate, which makes it impossible to clearly display the anatomical structure of the affected area. Compared with digital X-ray radiographs, MSCT postprocessing technology has a short scanning time and a fast speed [11, 12]. It has higher image resolution in both horizontal and vertical directions and will not affect overlap during the display of concealed fractures.

In order to improve the clinical detection rate of extremity bone and joint fractures, the hospital conveniently selected 80 cases of extremity bone and joint fracture patients treated from October 2019 to April 2020 as the research objects and compared with DR (DR). The diagnostic results of the postprocessing technology of slices and MSCT have achieved certain research results.

## 2. Methods and Materials

### 2.1. General Materials

80 cases of extremity bone and joint fracture patients admitted to the hospital were selected as the research object. The patient's fracture was mainly caused by traffic accidents, collisions, falls, and other factors. The number of males and females was analyzed. There were 44 males and 36 females. The age ranged from 27 to 59 years, with an average of (44.41 ± 1.26) years old. Traffic accidents, collisions, and falls were 21 cases, 29 cases, and 30 cases. Fracture location: limb and pelvic trauma were 58 cases and 23 cases. The specific conditions of 80 patients are shown in Figure 1.

### 2.2. Apparatus and Methods

All patients with bone and joint fractures of the extremities undergo digital X-ray plain film examination first, and the X-ray camera is provided by Philips. Then, we use MSCT to scan 80 patients with extremity bone and joint fractures. We use relevant operating instruments to adjust the patient's posture and posture to establish the correct scanning method.

In the process of CT scanning, the scanning range is divided. Position the fracture image of the patient and set the scan parameters reasonably. The control parameter is 120 kV, the reconstruction interval is 0.9 mm, the layer thickness is 5.1 mm, the reconstruction layer thickness is 1.26 mm, the bone window is osteo, and the reconstruction function is B80 svery sharp. Process the scanned data and reconstruct the image. According to the displayed surface shadow reorganization multiplane and three-dimensional imaging reconstruction technology, understand and master the multidirectional lesions of patients with extremity bone and joint fractures. The process of MSCT scanning fracture is shown in Figure 2.

### 2.3. Observation Indicators

We observe the fracture images of patients with limb bone and joint fractures, analyze the data of the patient's fracture lesions, understand and grasp the patient's fracture situation, and determine the types of limb bone and joint fractures. Finally, we made statistics on the detection rate of occult fractures of limbs and joints.

### 2.4. Statistical Methods

The statistical software SPSS18.0 was used to analyze the data in this study, using (*x* ± *s*) to represent measurement data and using the *t*-test method for comparison; using the test, percentage (%) represents counting data; when *P* < 0.05, the difference is statistically significant.

## 3. Results

### 3.1. Orthopaedic Imaging

Among 80 patients, 100 fractures were found. 22 cases of shoulder fractures included surgical neck fractures of the humerus with avulsion of the greater tuberosity, acromion of the clavicle of the shoulder joint with avulsion fractures of the humeral head, and scapular fractures. 17 cases of elbow joint fractures included humeral epicondyle fractures and radial head fractures, 21 cases of wrist joint fractures included scaphoid fractures and distal radius fractures, 14 cases of metacarpal base fractures, and 26 cases of hip fractures included iliac and acetabulum. Fractures can be combined with posterior dislocation of the femoral head, femoral neck, and intertrochanteric fractures.  Figure 3 shows DR plain film and MSCT images.

It can be seen from Figure 3 that the fractures shown on the DR film are all suspicious, while the MPR axis of the MSCT is conducive to the diagnosis of subtle fractures, and the image shows the separation of fracture fragments more clearly. Ilium, acetabulum, patella, ankle joint, posterior ankle, internal epicondyle of the humerus, and the base of the fourth and fifth metacarpal bones are easily misdiagnosed on DR digital radiographs due to overlapping images, small fracture lines, and no obvious misalignment. Using MSCT scan, which is then reconstructed by MPR, SSD, and VRT, the fracture image is clearly visible, especially the relationship between the fracture line, small fracture fragments, and adjacent tissue structures can be clearly displayed on multiple levels through MPR.

### 3.2. Comparative Results of Occult Fractures

We research and analyze the bone and joint fractures of the extremities, monitor the results of the X-ray detection data, analyze the abnormal detection of the X-ray, count the number of concealed fractures, and use the X-ray to detect the concealed fractures of the limbs and joints. There were 7 patients, and the detection ratio was 8.75%. Using MSCT postprocessing technology, 25 patients with occult fractures of limbs and joints were detected, with a detection rate of 31.25%. The difference of the detected data was compared, and the difference was obvious (*χ*^2^ = 12.1443, *P* < 0.05), which was statistically significant, as shown in Table 1.

DR examination of the ilium, acetabulum, posterior ankle of ankle, internal epicondyle of the homers, and the base of the 4th to 5th metacarpal bone overlaps, the fracture line is small, the dislocation is usually not obvious, and the misdiagnosis is easy to occur. In this case, using MSCT scanning to examine patients with occult fractures and then display surface shadows and reconstruction planes and reconstruct three-dimensional imaging, one can clearly observe the fracture images of patients with occult fractures, especially the reconstruction planes, which can be displayed on multiple levels. The upper will clearly show the patient's fracture line, relatively small fracture fragments, and the relationship between adjacent tissue structures.

### 3.3. Postprocessing Results of MSCT

The study showed that a total of 100 fractures were found in the enrolled patients, of which 69 fractures were found by DR examination, with a detection rate of 69%. After MSCT postprocessing technology inspection, MPR, SSD, and VRT found 96 fractures, 98 fractures, and 99 fractures, and the detection rates were 96%, 98%, and 99%. The paired test of the two inspection methods found that the accuracy of MSCT postprocessing technology in diagnosing limbs and joint fractures was significantly higher than that of digital X-ray. There was a statistically significant difference between linear photography and plain film (*P* < 0.05). The results of different methods of diagnosing joint injury types are shown in Figure 4.

## 4. Discussion

The MSCT scan speed is fast, and the image has high horizontal and vertical resolution [12, 13]. It shows that the hidden suspicious fracture has no image overlap with the X-ray plain film, and the image is clear. In this group of 80 patients, MPR can display fracture lines and bone fragments from any direction in two-dimensional cross-sectional, sagittal, coronal, oblique, and curved images on the display screen according to the needs of diagnosis, so as to have a more comprehensive understanding of the scope of fractures.

The three-dimensional effects of SSD and VRT are obvious [14–17]. Because SSD adopts threshold imaging, it is suitable for the display of the surface morphology of the skeletal system. It has a strong spatial three-dimensional effect and a clear surface anatomy relationship, which is conducive to the positioning of the fracture and the extent of the fracture line. The performance is obviously affected by the segmentation threshold in image processing, so the internal structure of the object cannot be displayed, and the density information of the object cannot be provided.

VRT uses all the voxel data of spiral CT volume scanning [18]. According to the CT value of each voxel and its surface characteristics, all voxels in the imaging volume are given different colors and different transparency through image reorganization and simulated light source illumination, as to show the full picture of organ or tissue structure with stereoscopic visual effect. VRT image can not only show the surface morphology of the observed object but also can display the morphology of any level inside the observed object according to the needs of the observer, helping to determine the bone and joint damage the main feature of the image of the positional relationship with the surrounding important structures is high resolution [19, 20]. It displays the density information while displaying the spatial structure to make up for the lack of SSD, but it is not as good as MPR in displaying the fine structure and small changes inside the fractured bone. SSD and VRT are inferior to MPR (patella fracture) when showing small fracture lines without obvious dislocation, and it is also inferior to MPR in terms of soft tissue damage and swelling [21]. MPR can better show the subtle and complex anatomical relationship between bone and joint damage and surrounding tissues and organs.

Due to the different fracture sites of the limbs and joints, the difficulty of detection is also greater, showing incremental and progressive changes. Among the bone and joint fractures of the extremities, occult fractures are difficult to diagnose. During the diagnosis process, many fracture problems are difficult to find as soon as possible, and omissions often occur, which are very detrimental to the rehabilitation of patients with bone and joint fractures [22]. This requires the determination of the principle of occult fractures and accurate determination and evaluation, so that the accuracy of clinical diagnosis can be effectively guaranteed. In diagnosing patients with bone and joint fractures of the extremities, although the use of X-ray films can be helpful, X-ray films have certain limitations in application. X-ray film limitation is very unfavorable for doctors to accurately judge the fracture status of limbs and joints in patients. The effective use of MSCT postprocessing technology is more advantageous than the application of X-ray film [23].

MSCT postprocessing technology not only has a fast-scanning speed but also has a very good scanning effect [24]. It can understand and master the vertical and horizontal changes of the scanned image and study and analyze the characteristics of the image. Suspicious fracture locations and hidden fracture locations are found and more in-depth assumptions and judgments of the symptoms of patients with limbs and joints. After the use of MSCT scanning, changes in the cross-section of the patient's limbs and joints will appear [25]. The cross-section, sagittal plane, coronal plane, and inclined plane are all planes. We distinguish the fracture line of the scanned image and understand the distribution of bone fragments in patients with limbs and joints. In this way, the range of fractures of limbs and joints in patients can be clearly defined. In the future, deep learning can be used for automatic diagnosis of patients and rehabilitation training through verification of external mechanical equipment [26–29]. After understanding the range of the patient's fracture range, research and analysis of the patient's soft tissue changes and accurately summarizes the data of the fracture of the limbs and joints. The mechanical information of such fractures are generally based on the material properties [30, 31].

## 5. Conclusion

Through the comparison of the detection results of occult fractures and the comparative analysis of the detection rate of fractures, it can be concluded that the postprocessing technology of MSCT is more advantageous than plain radiographs in judging the limbs and joints.

The use of MSCT postprocessing technology can detect the condition of the fractured parts of patients with extremity bone and joint fractures in a timely manner, effectively achieve clinical diagnosis, and have significant diagnostic results, so that the comprehensiveness and timeliness of treatment can be guaranteed. For patients with extremity bone and joint fractures, the staff can also give more accurate and comprehensive diagnosis results and use this as a basis to assist surgeons in formulating the corresponding fracture surgical treatment methods. At the same time, for patients with extremity bone and joint fractures, rehabilitation is also very helpful.

## Figures and Tables

**Figure 1:** The specific situation of 80 patients.

**Figure 2:** Flow chart of MSCT scanning fracture.

**Figure 3:** X-ray DR plain film and MSCT image.

**Figure 4:** The results of different methods to diagnose the type of joint damage.

**Table 1:** Comparative results of occult fractures of the two methods.

Method	Number of cases	Number of occult fractures	Proportion (%)
DR	80	7	8.75
MSCT	80	25	31.25
*χ* ^2^	12.1443		
*P*	0.02		

## Data Availability

The image data used to support the findings of this study have been deposited in the Musculoskeletal Radiographs (MURA) dataset (https://stanfordmlgroup.github.io/competitions/mura/).

## References

[1] Watson-Jones R. (1941). Fractures and other bone and joint injuries. *American Journal of Physical Medicine & Rehabilitation*.

[2] Laroche M., Ricq G., Cantagrel A. (1997). Bone and joint involvement in adults with Werner’s syndrome. *Revue du Rhumatisme*.

[3] Vardasca R., Restivo M. T., Mendes J. (2017). Skin temperature bilateral differences at upper limbs and joints in healthy subjects. *European Congress on Computational Methods in Applied Sciences and Engineering*.

[4] Kotsianos D., Rock C., Euler E. (2001). 3D imaging with a mobile surgical image enhancement equipment (ISO-C-3D). Initial examples of fracture diagnosis of peripheral joints in comparison with spiral CT and conventional radiography. *Der Unfallchirurg*.

[5] Urazgil'Deev Z. I., Roskidaĭlo A. S. (1999). Treatment of ununited fractures and pseudarthrosis of long bones of the lower limbs complicated by osteomyelitis. *Khirurgiia*.

[6] De-Xiang L. (2009). The application of anatomic locking compression plate in comminuted fractures of the limbs close to the joints about fracture patients. *Guide of China Medicine*.

[7] Coc I., Banic T., Bilic V. (2017). Neurological recovery after early reposition, decompression and instrumented fusion of C-type L2 fracture: a case report. *Global Spine Journal*.

[8] Hollinger A., Christe A., Thali M. J. (2009). Incidence of auditory ossicle luxation and petrous bone fractures detected in post-mortem multislice computed tomography (MSCT). *Forensic Science International*.

[9] Wedegärtner U., Gatzka C., Rueger J. M. (2003). Multislice CT (MSCT) in der Detektion und Klassifikation von Becken- und Azetabulumfrakturen. *RoeFo-Fortschritte auf dem Gebiete der Roentgenstrahlen und der Neuen Bildgebenden Verfahren*.

[10] Ronneberger O., Kainmueller D., Vorontsov E. (2009). The value of MSCT with three dimensional reconstruction in chest trauma fractures. *Journal of Medical Imaging*.

[11] Poudel R. P. K., Manish S., Montana G. (2015). The value of MSCT in the diagnosis of costae and costicartilage occult fractures. *Journal of Practical Medical Imaging*.

[12] Huaguo M. (2011). The diagnosis value of X-ray and MSCT in dislocation of scaphoid-lunate joint. *Journal of Mathematical Medicine*.

[13] Nigg B. M., Bae S. Y., Lee J. H. (2012). X-ray and MSCT in the diagnosis of severe spinal injury. *Image Technology*.

[14] Weinberg M. W., Davidson N. P. (2005). Clinical evaluation and diagnosis of 3D reconstruction and MPR with MSCT in tibial plateau fractures. *Journal of Medical Imaging*.

[15] Goyal A., Sharma S. (2013). Traumatic carotid-cavernous fistula: excellent demonstration on 3D CT angiography. *BMJ Case Reports*.

[16] Gang-Wei C., Wen-Bin M. U., Zheng-Yu J. (2013). Optic canal fracture evaluation using three-dimensional computed tomography reconstructions. *Medical Journal of Peking Union Medical College Hospital*.

[17] Jin W., Xue-Lin Z., Shu-Xiang L. I. (2003). Clinical application of spiral CT to acetabular fracture: surface shaded display (SSD) and volume rendering (VR) techniques study and compared with two-dimensional CT (2DCT), X-ray and MPR. *Journal of Practical Radiology*.

[18] Liu-Jin N., Guang-Yu L. I., Han-Hua P. (2013). Clinical significance of spiral CT with three-dimensional reconstruction imaging on palvic fracture. *Progress in Modern Biomedicine*.

[19] Shin W. J., Hastie G. R., Goodman D. A. (2000). Clinical applications of VRT 3D reconstruction with spiral CT. *Journal of Clinical Radiology*.

[20] Jankharia B., Sosi N. (2002). Radiology of acetabular fractures. *Indian Journal of Orthopaedics*.

[21] Weinberg M. W., Davidson N. P. (2000). Three-dimensional reconstructive imaging of electron beam CT: the clinical application and evaluation. *Bulletin of Medical Postgraduate*.

[22] Wolterink J. M., Pernu F., Pezold S. (2007). Application of three-dimensional reconstruction technique of 16 slice spiral CT for complicated fractures. *Journal of Rare and Uncommon Diseases*.

[23] Gerstenfeld L. C., Alkhiary Y., Krall E. A. (2006). Three-dimensional reconstruction of fracture callus morphogenesis. *Journal of Histochemistry & Cytochemistry Official Journal of the Histochemistry Society*.

[24] Liow R. Y. L., Birdsall P. D., Mucci B. (1999). Spiral computed tomography with two- and three-dimensional reconstruction in the management of tibial plateau fractures. *Orthopedics*.

[25] Kuroda T., Ikeuchi K., Nakade K. (2002). Three-dimensional reconstruction of cleavage fracture surface for duplex stainless steel. *Vacuum*.

[26] Huang L., Yin L., Liu B., Yang Y. (2021). Design and error evaluation of planar 2DOF remote center of motion mechanisms with cable transmissions. *Journal of Mechanical Design*.

[27] Bo H., Changjiang Z., Hongbing W., Lairong Y. (2021). Prediction and validation of dynamic characteristics of a valve train system with flexible components and gyroscopic effect. *Mechanism and Machine Theory*.

[28] Wong K. K. L., Fortino G., Abbott D. (2020). Deep learning-based cardiovascular image diagnosis: a promising challenge. *Future Generation Computer Systems*.

[29] Tang Z., Zhao G., Ouyang T. (2021). Two-phase deep learning model for short-term wind direction forecasting. *Renewable Energy*.

[30] Xinli X., Zhang C., Musharavati F., Sebaey T. A., Khan A. (2021). UFSW tool pin profile effects on properties of aluminium-steel joint. *Vacuum*.

[31] Xu X., Zhang C., Derazkola H. A., Demiral M., Zain A. M., Khan A. (2021). Dispersion of waves characteristics of laminated composite nanoplate. *Steel and Composite Structures*.

